The article "Apoptotic and Antioxidant Activity of Gold Nanoparticles Synthesized Using Marine Brown Seaweed: An In Vitro Study" was retracted in 2024. Reasons: signs of a paper mill; suspected computer-generated content; unreliable results or conclusions; concerns about the data.

# Apoptotic and Antioxidant Activity of Gold Nanoparticles Synthesized Using Marine Brown Seaweed: An In Vitro Study

**DOI:** 10.1155/2022/5746761

**Published:** 2022-07-13

**Authors:** S. Rajeshkumar, R. P. Parameswari, J. Jayapriya, M. Tharani, Huma Ali, Nada H. Aljarba, Saad Alkahtani, Saud Alarifi

**Affiliations:** ^1^Center for Transdisciplinary Research (CFTR), Nanobiomedicine Lab, Department of Pharmacology, Saveetha Dental College, Saveetha Institute of Medical and Technical Science, Saveetha University, Chennai, India; ^2^Department of Chemistry, Maulana Azad National Institute of Technology, Bhopal, India; ^3^Department of Biology, College of Science, Princess Nourah bint Abdulrahman University, P. O. Box 84428, Riyadh 11671, Saudi Arabia; ^4^Department of Zoology, College of Science, King Saud University, P. O. Box 2455, Riyadh 11451, Saudi Arabia

## Abstract

A major paradigm shift in the field of nanobiotechnology is the invention of an eco-friendly, economical, and green approach for synthesis of metal nanoparticles. In the present study, we have synthesized gold nanoparticles (AuNPs) using aqueous extracts of marine brown seaweed Sargassum longifolium. The synthesized nanoparticle was subjected to characterization using different techniques such as UV-Vis spectroscopy, Fourier transform infrared spectroscopy, atomic force microscope, scanning electron microscope, transmission electron microscope, and elemental dispersive X-ray diffraction. Further, the seaweed extract and the synthesized AuNPs were evaluated for its anticancer effect using MG-63 human osteosarcoma cells besides in vitro antioxidant effect. The formation of S. longifolium-mediated synthesis of gold nanoparticles was demonstrated by UV-Vis spectroscopy. Presence of elemental gold was confirmed by EDX analysis. TEM analysis demonstrated spherical morphology of the synthesized AuNPs and SEM analysis revealed the particle size to be in the range of 10-60 nm. The FTIR showed the presence of hydroxyl functional groups. The toxicity of S. longifolium extract and the synthesized AuNPs was tested using brine shrimp lethality assay at different concentrations with results showing both seaweed extract and AuNPs to be nontoxic. Both S. longifolium and AuNPs exhibited significant antioxidant activity by scavenging DPPH free radicals and H_2_O_2_ radicals. Significant antiproliferative effect was observed against MG-63 osteosarcoma cells. It was also shown that the seaweed extract and the AuNPs induced cytotoxicity in cell lines by mechanism of apoptosis. In conclusion, this study provided insight on AuNPs synthesized from S. longifolium as a potent antioxidant and anticancer agent.

## 1. Introduction

Nanotechnology has been defined as a field of study that integrates physics, chemistry, and biology principles to create new materials with unique features on a very small scale, referred to as the nanoscale (0–100 nm) [1]. It involves both research and technology, a new discipline of science and engineering [2]. Nanotechnology has pervaded practically every branch of science, allowing for the development of unique alternatives to many research tailbacks. Nanomedicine, a combination of nanotechnology and medicine offers various advantages over traditional treatment methods [3]. Metal nanoparticles have reinforced immense interest in the field of nanomedicine owing to their unique properties than their bulk counterpart [4]. However, the physicochemical methods adopted to produce these metal nanoparticles have intrinsic limits, which constitute a significant barrier to the science's maturity [5]. Therefore, development of eco-friendly technologies termed as “green approach” has found to be comparatively safe, nontoxic, inexpensive, and biocompatible [6]. During chemical formulation, there are high chances of contamination. Unlike other methods, green synthesis produces a pure form of NPs [7].

Due to their biocompatibility, low toxicity, ease of surface functionalization, and optical and electronic qualities, gold nanoparticles (Au-NPs) have sparked considerable interest than any other metal nanoparticles and hence utilized for various biomedical applications [8, 9]. Gold nanoparticles own the history of being used for various applications right from colouring glass to treating complex mental illness [10]. Moreover, the diverse fascinating properties of AuNPs, viz., electronic, magnetic, optical, and catalytic properties, have made AuNPs a suitable candidate for use in bioimaging like X-ray computed tomography, drug or gene delivery, diagnostic, therapeutics, tissue engineering, and theranostics [11, 12]. Further, AuNPs are prevalently used in the field of cancer therapy [13]. Despite possessing significant advantages, use of AuNPs has its own limitation due to application of various hazardous chemical synthesis methods for preparation. Hence, green synthesis method using plants, microbes, seaweeds, and its respective bioactive metabolites is used to synthesize AuNPs [14].

About 80% of the world's biodiversity has been found in the marine ecosystem. Among the various marine sources, seaweeds have gained immense response in different fields of research owing to its unique properties like high biodiversity, living habitats, and specific living conditions [15]. Seaweeds are found prevalent in harsh marine environment which possess numerous bioactive metabolites with various activities [16, 17]. Brown seaweeds are predominantly brown due to the presence of the carotenoid fucoxanthin and the primary polysaccharides include alginates, laminarins, fucans, and cellulose [17].

Sargassum species are tropical and subtropical brown macroalgae of the shallow marine meadow [18]. They are nutritious and rich sources of bioactive compounds such as vitamins, carotenoids, dietary fibers, proteins, and minerals [19]. Also, many biologically active compounds like terpenoids, flavonoids, sterols, sulphated polysaccharides, polyphenols, sargaquinoic acids, sargachromenol, and pheophytine were isolated from different Sargassum species [20]. These isolated compounds exhibit diverse biological activities like analgesic, anti-inflammatory, antioxidant, neuroprotective, antimicrobial, antitumor, fibrinolytic, immune-modulatory, anticoagulant, hepatoprotective, and antiviral activity. Hence, Sargassum species have great potential to be used in pharmaceutical and nutraceutical areas [21–23]. Several studies have exhibited the anticancer potential of Sargassum species studies against various tumour cells [24–27]. Similarly, AuNPs prepared using several other sources have been reported for its potent anticancer effect using liver cancer, lung cancer, and breast cancer cells [28–30]. Although many reports are available on the potential of Sargassum against various disorders, the green synthesized AuNPs mediated by the marine seaweed Sargassum longifolium have not been investigated. Therefore, in the present study, we synthesized Sargassum longifolium-mediated AuNPs and evaluated its antioxidant and anticancer effect.

## 2. Materials and Methods

### 2.1. Chemicals and Reagents

Gold (III) chloride trihydrate (HAuCl4·3H_2_O), 2,2-diphenyl-1-picrylhydrazyl, hydrogen peroxide (H_2_O_2_), MTT (3-(4,5-dimethylthiazol-2-yl)-2,5-diphenyltetrazolium bromide), ethidium bromide, and acridine orange were purchased from Sigma Aldrich, USA. Dulbecco's minimum essential media (DMEM), fetal bovine serum (FBS), penicillin/streptomycin, Trypsin-EDTA, phosphate buffered saline (PBS), and dimethyl sulfoxide were purchased from Gibco, USA. All other chemicals, reagents, and solvents used were of analytical grade and procured from Himedia, India.

### 2.2. Preparation of Extract

About 1 g of S. longifolium was mixed with 100 mL of double distilled H_2_O, boiled for 5 min, and filtered through Whatman No. 1 filter paper. It was refrigerated at 4°c for further experimental purpose.

### 2.3. Synthesis of AuNPs

To prepare the gold nanoparticles, 80 mL of aqueous sea weed extract was mixed with 20 mL of AuCl_4_ solution in a clean conical flask. The mixture was kept for stirring on a magnetic stirrer at room temperature. The change in the solution colour indicated the reduction of Au3+ ions in the solution, and the wavelength of which was measured at periodic intervals using UV-Vis spectrophotometer after the reaction reached saturation. Later on confirming the formation of AuNPs, the solution was centrifuged at 10,000 rpm for 15 min and pellet was collected for further analysis.

### 2.4. UV Visible Spectroscopy

The UV-Visible spectrum of the gold nanoparticles solution was recorded using double beam UV-Visible Spectrophotometer (UV-2450, Shimadzu). Optical density was taken from 360 to 650 nm (ranges increased 10 nm gradually) at different time points. Based on the OD values, the peak was identified and denoted as an optimum nanoparticles biosynthesis.

### 2.5. Microscopic Studies

A drop of sample was placed on carbon-coated copper grid, air dried at room temperatures, and stained with 2% uranyl acetate. The nanoparticle size measurement was done using transmission electron microscope (Hitachi, H-7500), and average nanoparticle size was considered as the size of the sample. The morphological characterizations of the S. longifolium were performed using SEM. To know the exact particle size and nanosize effect, the sample was characterized using atomic force microscope (AFM), which measures the atomic range of the particle.

### 2.6. FTIR

FTIR measurements demonstrate the presence of functional groups which can be liable for capping leading to proficient stabilization of the gold nanoparticles. The refined suspension containing the nanoparticles was completely dried and ground with KBr pellets and used for FTIR analysis. In order to obtain decent signal/noise ratio, 512 scans were verified to get appropriate results.

### 2.7. EDX

Energy dispersive X-ray spectroscopy is a technique used for determination of elemental analysis of S. longifolium. It can be used to basically determine the amount of AuNPs produced with a thin film of bacterial biomass.

## 3. Antioxidant Activities

### 3.1. DPPH Free-Radical Scavenging Assay

The free-radical scavenging activity of the biosynthesized gold chloride nanoparticles and the S. longifolium extract was evaluated by DPPH free-radical scavenging assay. The seaweed extract, seaweed extract-mediated gold nanoparticles, and standard ascorbic acid were prepared at different concentrations of 2-10 *μ*g/mL.1 mL of different concentration seaweed extract, AuNPs, and standard to appropriately labelled test tubes. To the above test tubes, 1 ml of 0.1 mM DPPH prepared in methanol and 450 *μ*L of 50 mM Tris HCl buffer (pH 7.4) were mixed and incubated in dark for 30 minutes.1 mL of distilled water, 1 ml of DPPH, and 450 *μ*l of 50 mM Tris HCl buffer served as control blank. The absorbance of the solution was measured at 517 nm. The percentage inhibition of free radical formation was determined from the following equation:

(1) $$\begin{array}{c} \%\text{inhibition}=\frac{\text{Absorbance of control}-\text{absorbance of test sample}}{\text{Absorbance of control}}\times 100. \end{array}$$

### 3.2. Hydrogen Peroxide Scavenging Assay

The H_2_O_2_ radical scavenging activity was determined for the S. longifolium extract, AuNPs. Different volume (10 *μ*L-50 *μ*L) of S. longifolium extract and AuNPs were added to appropriately labelled test tubes and incubated with 50 *μ*L of 5 mM H_2_O_2_. Ascorbic acid served as standard reference. Blank control consisted of 50 *μ*L of 5 mM H_2_O_2_ devoid of the sample. The test tubes were allowed to incubate for 20 min at room temperature. The absorbance was measured at 610 nm. The percentage inhibition of H_2_O_2_ radical formation was determined from the following equation:

(2) $$\begin{array}{c} \%\text{inhibition}=\frac{\text{Absorbance of control}-\text{absorbance of test sample }}{\text{Absorbance of control}}\times 100. \end{array}$$

### 3.3. Brine Shrimp Lethality Assay

2 g of iodine free salt was weighed and dissolved in 200 mL of distilled water in which dried cysts were placed. The larvae (nauplii) were hatched after 36 h of incubation under conditions of strong ventilation and continuous illumination. The evaluation of cytotoxicity was carried out using nauplii of brine shrimp as follows: Briefly, 5 ml of water was filled in 6 well ELISA plates. Fresh suspensions of S. longifolium extract and AuNPs were prepared using the artificial sea water at 1-fold serial dilution between the range of 10 *μ*L, 20 *μ*L, 30 *μ*L, 40 *μ*L, and 50 *μ*L. The different concentration seaweed extract and the synthesized AuNPs were added to the 6-well plates. To that 10 nauplii were slowly added to each well, and the plates were incubated for 48 h. After every 24 hours, the ELISA plates were observed for number of live nauplii's using stereoscopic microscope and the lethality was calculated using following formula: %lethality = (number of dead nauplii)/(number of dead nauplii + number of live nauplii) × 100.

### 3.4. Cell Culture

Human osteosarcoma cell line MG-63 was purchased from National Centre for Cell Sciences (NCCS), Pune with the passage number of 16. The cells were grown in Dulbecco's modified Eagle medium (DMEM) supplemented with 10% fetal bovine serum (FBS), 100 U/mL penicillin, and 100 U/ml of streptomycin at 37°C in 95% humidified air with 5% CO_2._ On reaching 80-90% confluency, the cells were trypsinized using 0.25% Trypsin-EDTA and plated for further assays.

### 3.5. Anticancer Activity–MTT Assay

The cytotoxic potential of the synthesized gold nanoparticles was assessed on human osteosarcoma cell lines, MG-63. Briefly, cells were grown in 96-well plates at a density of 5 × 10^4^ cells/well. After 24 h of incubation, the cells were treated with different concentrations (1, 5, 10, 20, 40, and 80 ng/mL) of the seaweed extract and the synthesized gold nanoparticles. Cells which did not receive treatment with either seaweed extract or gold nanoparticles, were treated as controls. After 24 h of incubation, media was aspirated from all the wells and 50 *μ*l of MTT (3-(4,5-dimethylthiazol-2-yl)-2,5-diphenyltetrazolium bromide) was added at a concentration of 5 mg/mL prepared in PBS (phosphate buffered saline). After 4 h of MTT incubation, 150 *μ*L of DMSO (dimethyl sulfoxide) was added to dissolve the purplish formazan product. Absorbance was read at 540 nm using Multimode reader (Perkin Elmer, USA). The % inhibition of cell proliferation was calculated using the following formula: ((OD of control − OD of the test)/OD of the control)∗100.

### 3.6. Dual Ethidium Bromide/Acridine Orange (EtBr/AO) Staining Assay

AO/EtBr staining of MG-63 cells was performed as per Banda et al. [31]. MG-63 cells 4 × 10^5^/well were treated with two different concentrations of seaweed extract (16 and 32 ng/ml) and c (12 and 24 ng/mL) for 24 h. The concentrations for apoptosis assay were selected based on IC_50_ value. After 24 h, the media was aspirated. The cells were stained using AO/EtBr dual staining solution prepared in PBS by incubating the cells with 5 *μ*L of a mixture of AO/EtBr (60 *μ*g/mL (acridine orange)/100 *μ*g/mL (ethidium bromide)) for 5 min in the dark after staining. The cells were immediately imaged in a fluorescence microscope (Nikon Eclipse E200, Tokyo, Japan).

## 4. Results and Discussion

### 4.1. Biosynthesis of AuNPs and UV-Vis Spectroscopy

Aqueous extract of S. longifolium was added into gold chloride solution. The formation of AuNPs was confirmed by the development of colour which is characteristic of AuNPs. The confirmation was done by recording the UV-Vis absorbance was at 350-650 nm which corroborated with the earlier published results [14, 32] in which the UV-Vis spectral analysis of AuNP absorbance was measured at 520-560 nm (27). They confirmed the peak around 540 nm and a broader peak between 700 and 800 nm.

### 4.2. Microscopic Analyses

The results of SEM and TEM revealed the size and shape of AuNPs, respectively (Figures 1 and 2). SEM analysis exhibited uniformly distributed AuNP which was found to be spherical in morphology with size ranging between 10 and 60 nm. Some of the AuNPs were seen aggregated. The separation between nanoparticles was observed from TEM image due to the presence of capping agent. The images of AFM showed the presence of AuNPs synthesized by S. longifolium (Figure 3). From the images, it is confirmed that a nanoplate structure was formed proving this method to be appropriate and successful for the synthesis of AuNPs [27].

### 4.3. FTIR

The functional groups of the S. longifolium-synthesized gold nanoparticles are shown in Figure 4. FTIR shows the characteristic peaks indicating the presence of different functional groups. A broad band observed at 3265 cm^−1^ was shown to be associated with C-H and O-H stretches from carboxylic acids and alcohols. The carboxylic group assigned at 1232 cm^−1^ corresponds to C-O stretch, presence of amides, and N-H stretch at 1608 cm^−1^. The analysis also revealed the presence of nitro groups N=O stretch at 1506 cm^−1^. Other weak band also present at 455 cm^−1^ corresponds to alkyl halides.

### 4.4. EDX Analysis

EDX was performed to analyse the presence of various elements in the synthesized AuNPs. In Figures 5(a) and 5(b), a strong atomic signal from Au atom was observed with atomic % of 3.50% along with O atom 22.12%, C atom 69.56%, K atom 1.89%, and Cl atom 2.93%; there were no evident peaks for other elements or impurities [32].

### 4.5. Toxicological Evaluation of S. Longifolium Extract and Its Synthesized AuNPs

Figure 6 shows the brine shrimp lethality assay, and it is a preliminary and important screening tool to evaluate the toxicity of a drug. In the cytotoxic effect, the percentage of live nauplii was calculated. On day 1, the different concentrations of synthesized AuNPs as well as control showed 100% live nauplii. On the 2^nd^ day except 40 *μ*L and 50 *μ*L, other concentrations exhibited 100% survival which was in comparison to that of untreated control. Minimum lethality (20%) was observed in 40 *μ*L and 50 *μ*L AuNP-treated groups on day 2. From the results, the nontoxic nature of the synthesized AuNPs was inferred up to 30 *μ*L towards brine shrimps [7].

### 4.6. DPPH Free-Radical Scavenging

The antioxidant activity of formulated AuNPs and the seaweed extract was estimated by evaluating the percentage inhibition of DPPH radicals (Figure 7). The DPPH radical scavenging activity of AuNPs was found to be directly proportional to the concentration of the seaweed extract and its synthesized AuNPs. The results exhibited significant inhibition of DPPH free radicals in a dose-dependent manner at 10, 20, 30, 40, and 50 mg/ml. AuNPs showed marked radical scavenging activity when compared to seaweed extract. The results revealed that the AuNPs were found to be more potent than the seaweed extract which was comparable with that of standard ascorbic acid [7].

### 4.7. H_2_O_2_ Radical Scavenging Activity

The H_2_O_2_ scavenging effect of S. longifolium extract and its mediated synthesis AuNPs was found to be dose-dependent (Figure 8). The free radical scavenging ability of the seaweed extract and the AuNPs was compared to standard ascorbic acid. AuNPs exhibited better scavenging effect than seaweed extract alone [5].

### 4.8. Anticancer Activity

#### 4.8.1. Cytotoxicity Evaluation by MTT

The cytotoxicity activity of S. longifolium extract and its synthesized AuNPs was determined using MG-63 human ostoesarcoma cells by MTT assay (Figure 9). The results showed dose-dependent cytotoxic effect of both seaweed extract and AuNPs. A maximum inhibition of 72.5% was observed in seaweed extract whereas the AuNPs showed 81.5% inhibition at higher concentration of 80 ng/ml indicating that the seaweed-synthesized AuNPs is more potent than seaweed extract alone. The IC_50_ was found to be 32 ng/ml for seaweed extract and 23.58 ng/ml for AuNPs, respectively. Earlier published data have reported that AuNPs induce cytotoxicity by means of oxidative stress which results in production of reactive oxygen species thereby causing impairment in mitochondria function, ultimately resulting in cell death [33, 34].

#### 4.8.2. Apoptosis Assay by EtBr/AO Dual Staining

MG-63 cells were treated with seaweed extract and AuNPs. After 24 h incubations, the cells were stained using EtBr/AO dual stain and the morphological changes were observed by examining under fluorescent microscope. Dual staining of the treated and control cells demonstrated induction of apoptosis by the seaweed extract and AuNPs. Viable cells emitted green fluorescence while early and late apoptotic cells appeared yellowish orange and orange in colour (Figure 10). Red fluorescence indicates necrosis. Previously published data has demonstrated that oxidative stress triggers apoptosis by activation of p38 MAPK pathway (34). In line with this, the present study findings have shown that the synthesized AuNPs might have induced apoptosis by oxidative stress-mediated pathway. However, further studies are needed to elucidate the mechanism of action.

## 5. Conclusion

In this present study, we have reported an eco-friendly method for green synthesis gold nanoparticle synthesized from marine seaweed S. longifolium. The results demonstrated the presence of elemental gold. Both seaweed extract and AuNPs exhibited significant free-radical scavenging activity indicating that they possess antioxidant effect. Also, the nontoxic nature of AuNPs was also confirmed by brine shrimp lethality assay. The cytotoxic and apoptotic effect of the AuNPs was also confirmed in MG-63 cell line which might be due to induction of oxidative stress in the MG-63 cells. However, in vivo and molecular studies are warranted in future to elucidate the exact mechanism of anticancer effect rendered by S. longifolium-mediated synthesized AuNPs.

## Figures and Tables

**Figure 1:** Representative SEM images of (a) S. longifolium and (b) its mediated gold nanoparticles.

**Figure 2:** Representative TEM images of S. longifolium and S. longifolium-mediated gold nanoparticles (scale-200 nm).

**Figure 3:** Representative AFM images of S. longifolium-mediated gold nanoparticle.

**Figure 4:** FTIR spectrum of S. longifolium-synthesized gold nanoparticles.

**Figure 5:** (a) EDX spectrum S. longifolium-mediated gold nanoparticle; (b) the elements, its weight %, and atomic %.

**Figure 6:** Effect of S. longifolium and its mediated gold nanoparticle represented as % of nauplii on day 1 and day 2.

**Figure 7:** % inhibition of DPPH free radicals by AuNPs mediated from S. longifolium and S. longifolium extract. Results are expressed in terms of mean ± SEM (*n* = 3).

**Figure 8:** % inhibition of H_2_O_2_ free radicals by AuNPs mediated from S. longifolium and S. longifolium extract. Results are expressed in terms of mean ± SEM (*n* = 3).

**Figure 9:** Representative graph demonstrating the antiproliferative effect of S. longifolium and its synthesized AuNPs determined by MTT assay. Results are expressed in terms of mean ± SEM (*n* = 3).

**Figure 10:** Induction of apoptosis by seaweed extract and its mediated synthesis AuNPs. (a) Untreated control; (b) seaweed extract 16 ng/ml; (c) seaweed extract 32 ng/ml; (d) AuNPs 12 ng/ml; (e) AuNPs 24 ng/ml. Magnification: 20x.

## Data Availability

The research data used to support the findings of this study are included within the article.
